# Classification of Bioinformatics EEG Data Signals to Identify Depressed Brain State Using CNN Model

This article has been retracted.

**DOI:** 10.1155/2022/5214195

**Published:** 2022-04-13

**Authors:** Anuradha Thakare, Manisha Bhende, Nabamita Deb, Sheshang Degadwala, Bhasker Pant, Yekula Prasanna Kumar

**Affiliations:** ^1^Department of Computer Engineering, Pimpri Chinchwad College of Engineering, Pune, India; ^2^Marathwada Mitra Mandal's Institute of Technology, Pune, India; ^3^Department of Information Technology, Gauhati University, Assam, India; ^4^Department of Computer Engineering, Sigma Institute of Engineering, India; ^5^Computer Science & Engineering, Graphic Era Deemed to Be University, Dehradun, Uttarakhand, India; ^6^Department of Mining Engineering, College of Engineering and Technology, Bule Hora University, Blue Hora, 144 Oromia Region, Ethiopia

## Abstract

Patients suffering from severe depression may be precisely assessed using online EEG categorization and their progress tracked over time, minimizing the risk of danger and suicide. Online EEG categorization systems, on the other hand, suffer additional challenges in the absence of empirical oversight. A lack of effective decoupling between brain regions and neural networks occurs during brain disease attacks, resulting in EEG data with poor signal intensity, high noise, and nonstationary characteristics. CNN employs momentum SGD optimization. By using a tiny momentum decay factor, the literature's starting strategy, and the same batch normalization, this work attempts to decrease model error. Before being utilized to form a training set, samples are shuffled, followed by validation and testing on the new samples in the set. An online EEG categorization system driven by a convolution neural network has been developed to do this. The approach is applied directly to the EEG input and is able to accurately and quickly identify depressed states without the need for preprocessing or feature extraction. The healthy control group and the depression control group had accuracy, sensitivity, and specificity of 99.08 percent, 98.77 percent, and 99.42 percent, respectively, in experiments on depression evaluation based on publicly accessible data. The machine learning technique based on feature extraction is often getting more and more complex, making it only suited for offline EEG categorization. While neural networks have become increasingly important in the study of artificial intelligence in recent years, they are still essentially black-box function approximations with limited interpretability. In addition, quantitative study of the neural network shows that depressed patients and healthy persons have remarkable dissimilarity between the right and left temporal lobe brain regions.

## 1. Introduction

Online EEG categorization has thrived as a critical component of brain health services for remote monitoring and assessment of brain illnesses such as epilepsy [1] and depression (MDD) [2]. Accurate evaluation of the brain's health and early surveillance of its growth can help limit the risk of danger [3]. EEGs are typically intense noise and nonstationary activity, and their accurate classification remains a critical issue [4]. It has been involved in two areas of study for decades: (1) preprocessing and (2) extraction of features. Preprocessing is used to reduce noise and false inverses from electroencephalogram (EEG) recordings. The electroencephalogram categorization has long been the focus of neuroscience research and therapeutic treatment. Machine learning approaches have risen in popularity over the years, and the majority of active research is concentrated on feature extraction. The disturbance and interference are almost always integrally related to the patient, and eliminating them, even if theoretically conceivable, necessitates time-consuming manual processing. In most cases, noise and interference are intrinsically linked to the patient, and removing them, even if theoretically possible, requires costly manual processing [5]; feature extraction enables dimension reduction and facilitates feature extraction.

It facilitates the efficient exploration of potentially interesting signals [6]. In recent years, time-frequency analysis has achieved an accuracy of 87.5 percent when used as the primary approach for EEG feature extraction [7]. Not only are traditional preprocessing and feature extraction approaches computationally intensive but their classification performance continues to fall short of the increasing accuracy requirements of clinical practice applications.

Classification of the electroencephalogram has long been a focus of neuroscience research and clinical practice. The majority of current research is focused on feature extraction, and machine learning techniques have exploded in popularity in recent years. The leading position in this direction is as follows: The literature [8] proposed a classification method based on wavelet transform-based time-frequency decomposition that had an 87.5 percent diagnostic accuracy for MDD patients and healthy controls. To efficiently detect the diverse lesions associated with severe depression, a technique for extracting spectral-spatial features from EEG data was devised, which attained an average accuracy of 81.23 percent [9]. Convolutional neural networks (CNN [10]) appear to have an edge over classic classifiers such as support vector machines when it comes to identifying noisy data. The conventional neural network is very simple to comprehend and execute. It anticipates photos with the highest classification of any algorithm. The fundamental benefit of CNN over its forebears is that it discovers essential traits with no need for human interference. The “data recorder” character, higher computing cost, proclivity for classifier, and experimental character of model construction are all drawbacks. They have shown success in detecting epilepsy [1] and Parkinson's illness [11]. Sufficient performance has been achived while maintaining a high level of noise immunity [12]. Feature extraction-based machine learning is typically computationally intensive and is therefore only suitable for offline EEG classification.

While neural networks have played a critical role in the field of artificial intelligence in recent years, they are merely black-box function approximates with little interpretability. It is a huge challenge to determine and comprehend if a neural network is producing accurate predictions [13]. When AI systems are simple to comprehend, they can assist in making better judgments, improving model design, generating more relevant discoveries, and increasing trust in AI. The major goal of mental wellbeing Ai technologies is to investigate the links across preventative or possible treatments and health experience. Diagnoses, medication research, personalized medicine and patients management of chronic conditions are all the areas where AI systems are used. Using depression as an example, a system is judged acceptable while neural network generates proper categorization by recognizing main elements that describe the brain disorder. On the contrary, despite the right placement of the end product, the neural network does not assess the critical qualities. Nevertheless, peripheral variables are determined as a result of the accurate detection of noise or interference. Due to an overwhelming number of false positives, this neural network cannot fulfill medical criteria. As a result, it is vital to decouple the neural network black box when brain disorders develop by assessing the complicated link between brain areas and models. In comparison to previous research, this study intends to develop a system that can (1) accurately classify raw EEG signals live, (2) ease the effort associated with preprocessing and feature extraction, and (3) give quantitative explanations using a neural network.

This research paper is organized into five sections: The introduction is describe in Section 1, proposed CNN Model is describe in Section 1.1, Section 2 describes environmental setup and result analysis, and finally, conclusion is describe in Section 3.

The contributions of this paper are as follows:

- Design and implement an online EEG signal classification platform based on cloud services. The platform takes a CNN as the core, the model is trained on the cloud server, and the hot deployment and online classification tasks are implemented on the local gateway
- A method based on AP clustering information entropy is proposed to realize the quantitative analysis service of the classifier model and realize the decoupling of the neural network black box

### 1.1. Proposed CNN Model

This paper first introduces the system architecture shown in Figure 1 and then discusses the design of the CNN and the core component of the system.

The gateway receives the EEG time slice first. The gateway then primarily handles model download and data upload operations in response to user requests. After obtaining the most recent learned classifier from the cloud, the gateway uses hot deployment to load it into the gateway. The EEG segments are then classified immediately, with the classification findings presented on appropriate intelligent devices such as desktop computers and smart phones. Following that, the doctor calibrates and uploads the user's permitted EEG data to the cloud server. Finally, the cloud server will train the model progressively. Following evaluation of the trained model by the administrator, the associated classifier model file is stored for download by the gateway.

### 1.2. CNN Based on a Cloud Computing Platform

The Internet of Things may take use of scalable and on-demand storage and processing provided by cloud computing systems. The classifier is trained and evaluated as part of cloud maintenance.

#### 1.2.1. CNN Network Structure

As seen in Figure 2, the architecture of a CNN that utilizes the fewest hidden layers feasible while still performing well in classification is illustrated. Dropout layers are followed by convolution layers, a max-pooling layer, and three fully connected layers. A Bayesian hyperparameter optimization procedure is used to optimize the model's hyperparameters. The parameter structure for convolution layer is as follows: There are a number of filters at (receptive field size), and the sigmoid activation functions of all completely connected layers FC are presented. This research tries to reduce model error by using a tiny velocity decay factor, the literature's starting strategy, and the same convolution layers; this work attempts to decrease model error. Before being employed to form a training set, samples are shuffled, followed by validation and testing on the new samples in the set. A 5-fold cross-validation approach was used to test the training and validation set classifiers.

The categorization results for a certain EEG time slice are generated using the CNN's final sigmoid activation function. The following is a summary of the most important design considerations:

- For high-dimensional raw EEG segments, the “high convolution layer” uses a large number of convolution filters, each filter only processing one channel of data on a single convolution layer. In order to structure the whole segment as a channel-stacked 3D data block for each time frame, the time-series data (1 024) from each electrode will be reshaped into a square matrix (32 32).
- The “Hourglass” FC layer block was designed in order to quickly reduce the number of neurons and model parameters. The building's construction has many FC levels. The input layer is closer to the output layer when there are fewer neurons in the output layer. Finally, in this study, the “hourglass” shape is formed by the last three completely connected (FC) layers

#### 1.2.2. Model Training and Testing

Momentum SGD optimization is used by CNN. This study tries to reduce model error by employing a small momentum decay factor [14], the literature's initialization approach [15], and the same batch normalization [16]. Samples are shuffled before being used to create a training set, followed by validation and testing on the new samples in the set. Training and validation set classifiers were tested using a 5-fold cross-validation method. The classification performance of the test set has been reported. These parameters are then fine-tuned via back propagation training [14].

(1) $$\begin{array}{c} \left\{\begin{array}{c} v_{i+1}⟵0.9.v_{i}-0.0001.\epsilon .w_{i}-\epsilon {\left(\frac{dL}{dw}\left|w_{i}\right.\right)}_{D_{i}}\\ w_{i+1}⟵w_{i}+v_{i+1} \end{array},\right. \end{array}$$

where *i* is the number of iterations, *v* is the momentum variable, *ε* is the learning rate, and (*dL*/*dw*|*w*_*i*_)_*D*_*i*__ is the partial derivative of the objective function concerning the connection weight *ω* on the *D*_*i*_ batch, which shows the optimization direction of the current collection.

The model may be tested on the test set once it has been trained (or new EEG time slices). It is flattened into a vector after a dropout layer, two convolution layers, and a one-to-one mapping layer. After that, the vectors pass via the FC layers with output sizes of 300, 60, and 1, before exiting the pipeline. Finally, the status of the EEG is shown.

EEG data from the gateway is downloaded and used to train the current model on the cloud server. In either case, the classification performance will either become better or worse. If a classifier's efficiency is reduced by more than 1%, it will be removed from service.

### 1.3. Complexity Explanation of CNN

This section primarily discusses the input layer's activation maximization. The depiction of the underlying neurons' characteristics provides a network's comprehensive picture. While the network seldom employs neurons in isolation, comprehension remains personal. To this end, we hope to verify the model's rationality and increase the objectivity of the explanation by measuring the information entropy of the input pattern.

#### 1.3.1. Activation Maximization

The input pattern with the greatest significant activation value for a certain hidden layer unit is identified by maximizing activation values. A linear activation function for the first layer's nodes means the first layer's input pattern is directly proportional to the filter's definition.

(2) $$\begin{array}{c} x^{*}=\arg\underset{x:t,\left|\left|x\right|\right|=\rho }{\max}\left(h_{ij}\left(\theta ,x\right)-\lambda \left(x\right)\right). \end{array}$$

There are three of these: *h*_*ij*_(, *x*), which represents the activation value of the *j*th layer of the neural network's *i*th neuron; *h*_*ij*_, which represents a function that combines input *x* with the model parameter; and (*x*), which represents input *x* as a standard term. The goal should be to activate *x*∗ as much as possible. This optimization problem is often nonconvex since *h* is not a specific function. It is possible to estimate the issue using gradient descent, which involves finding a local minimum, calculating *h*_*ij*_(, *x*) and then moving *x* in the direction of *h*_*ij*_(, *x*):

(3) $$\begin{array}{c} \frac{\partial h_{ij}\left(\theta ,x\right)-\lambda \left(x\right)}{\partial x}. \end{array}$$

A predetermined threshold is crossed when the amount of moving *x* falls below a certain level, signaling convergence. Because the classifier's first layer is determined, the activation maximization value is used to define the neural network's activation pattern. There are twenty matrices for each channel's ideal activation characteristic, which are recorded in terms of the channel's size (20 × 32 × 32) and computed as twenty activation tables.

#### 1.3.2. Information Entropy-Based on Neighbor Propagation Clustering

The primary function of information is to eliminate the complexity of things, and entropy information shows the unpredictability and information complexity

(4) $$\begin{array}{c} H\left(X\right)=-\underset{x\in X}{\sum }p\left(x\right)lbp\left(x\right), \end{array}$$

where *X* is a random variable and *p* (*x*) is the probability of random variable *X*.

The information entropy estimated by two distinct partitions is depicted in Figure 3. The data associated with the same partition will be categorized into the appropriate section, and the information entropy will be determined using formula (4). The distinction is that the conventional approach assumes that brain data follows a uniform distribution and is separated into equal distances (in Figure 3(b), the data is divided into six equal parts). When sufficient data sample points are available, the calculated results will be close to reality, but when there is insufficient, the error associated with this equidistant calculation of entropy is relatively large, and the uncertainty relationship of random variables cannot be measured effectively. Simultaneously, the clustering division takes the sequence's difference into account. It is an effective division (in Figure 3(a), due to the data distribution, the difference is divided into three parts, and the division interval of each piece is different). The data's features are given in detail to allow for an accurate computation of information entropy. All activation matrices are mapped to brain channels once their entropy is determined.

#### 1.3.3. AP Clustering Algorithm

Clustering by Proximity Propagation (AP) [17] is a clustering approach that is based on the flow of information between data points. The standard cluster analysis approach does not require a priori knowledge of the number of clusters. Rather than that, it keeps the greatest clustering performance by iterating through each sample point's contending cluster centers.

The similarity between sample data *s* [*i*, *j*] (*i*, *j* = 1, 2, ⋯, *N*) is used as the input to the AP clustering algorithm. The Euclidean distance is used in this research to represent the element value in the similarity matrix *S*. The diagonal element of *S* is a reference matrix *P*, which represents the likelihood of each sample point being chosen as the division centre. The AP algorithm iteratively traverses the sample data, constructing the responsibility matrix and the availability matrix, until it identifies a suitable cluster center *xk*; the iterative formula is as follows:

(5) $$\begin{array}{c} \left\{\begin{array}{c} R\left(i,k\right)⟵S\left(i,k\right)-\underset{k^{\prime }s.t.k^{\prime }\neq k}{\max}\left\{A\left(i,k^{,}\right)+S\left(i,k^{,}\right)\right\}\\ A\left(i,k^{.}\right)⟵\min\left\{0,R\left(k,k\right)+\underset{i^{,}s.t.i^{,}\notin \left(i,k\right)}{\sum }\max\left\{0,R\left(i^{,},k\right)\right\}\right\} \end{array}.\right. \end{array}$$

In comparison to the *K*-means method, this method has the following advantages: (1) no need for artificial initial cluster centers; (2) cluster centers are actual data samples, not virtual new data samples; (3) it is not sensitive to the initial value; and (4) the result's squared error is negligible.

#### 1.3.4. Information Entropy of Data Partitioning Based on AP Clustering

Three stages comprise the calculation of information entropy (APM) for data partitioning based on AP clustering. To begin, the signals *X* are sorted (in ascending order) to accelerate AP clustering convergence. Second, split the variables using the AP clustering technique and extract the coordinates of the highest (*Z* maxi) and minimum (*Z* mini) values for every partition *i*. The partition center *C*_*i*_ and its associated partition radius *R*_*i*_ are determined as follows (*Z* denotes the partition center's coordinates):

(6) $$\begin{array}{c} C_{i}=\frac{Z_{\max}^{i}+Z_{\min}^{i}}{2},R_{i}=\frac{\left|Z_{\max}^{i}-Z_{\min}^{i}\right|}{2},s.t.Z\in X,Y. \end{array}$$

Given two partitions *P*_*i*_ and *P*_*j*_, the demarcation point should be:

(7) $$\begin{array}{c} D\left(i,j\right)=\frac{\left(C_{j}-R_{j}\right)-\left(C_{i}+R_{i}\right)}{2},s.t.j>i. \end{array}$$

After the data division is obtained, the corresponding probability is accepted for the data falling into different divisions, and then, the information entropy of the sequence is obtained. The characteristics of the data are described in great detail to allow for a precise estimation of information entropy. Once the entropy of all activation matrices has been calculated, they are mapped to brain channels. The entropy information method would be calculated using the formula, and the data associated with the same partition will be grouped into the appropriate section.

To characterize the complex relationship between brain regions and models, first, obtain the maximum activation feature each channel's matrix (see Section 1.2.1) and then flatten all the matrices into a sequence to calculate its data partition entropy-based information on AP clustering; the entropy's information is projected as the complication at the channel level, and then, the brain regions are divided according to the 10-20 international EEG system (Table 1). Finally, the average value of the complexity within the brain region is calculated as the complexity between the brain region and the model.

## 2. Experimental Setup and Result Analysis

### 2.1. Data Description

EEG data from patients with severe depression and healthy controls are included in the public dataset [8]. The study also included a healthy control group, which was not subject to any mental or physical illness. First twenty electrodes of the EEG sensor were included in the data set, which was calibrated at 256 Hz using the International System 10-20. The sample space was divided into 18442 pieces (time slices for depression: 9789 and time slices for health: 8653).

### 2.2. Computational Complexity

The test setting for this experiment consists of an Intel i7 CPU operating at 3.33 GHz, 24 GB of RAM, and a 64-bit Windows 7 personal computer. The suggested classifier in this article is based on a subconvolutional neural network and a partially connected neural network. The temporal complexity of subconvolutional neural networks is first discussed. Its complexity in terms of time is related to the number of network layers (*L*) and their associated hidden neurons (*N*). The following formula is used to determine the temporal complexity of the full subconvolutional neural network:

(8) $$\begin{array}{c} O\left(S\left(N,L\right)\right)=O\left(\overset{d}{\underset{l=1}{\sum }}n_{l-1}.s_{l}^{2}.n_{l}.m_{l}^{2}\right). \end{array}$$

In the *l*th layer, the index is *l*, and the depth is *d*; *nl* is the number of filters (also known as width) and *nl* − 1 is the number of input channels in the *l*th layer, and finally, the spatial filter size (*sl*) and the output feature map size (*ml*) are the two parameters that represent the *l*th layer's depth (feature map).

For the subfully connected neural network, assuming the network has *L* layers, each layer has *U* neurons, and the classifier's time complexity is *O*.(*UL*). As a result, CNN's computational complexity is *O* (*S*(*N*, *L*)) + *O*.(*UL*).

### 2.3. The Influence Experiment of the Optimizer

This section compares several CNN optimization approaches, such as our momentum SGD, RMSprop [18], Adagrad [18], Adadelta [18], Adam [18], Adamax [18], and Nadam [18]. As seen in Figure 4, SGD obtains the greatest performance in this investigation, while the three optimization approaches (Adagrad, Adam, and Nadam) perform badly. The Adagrad approach modifies the corresponding learning rate for each parameter in each time step in accordance with previously determined parameter gradients. Local minimum and poor performance, the Adadelta technique is an extension of Adagrad that addresses the learning rate decay issue and improves performance. In this article, momentum-based approaches such as momentum SGD and RMSprop optimization are used to optimize the magnitude of the skip function during the training phase; that is, the local optimal point can be skipped. While Adam-based optimization methods such as Adam, Adamax, and Nadam are designed to rapidly train neural networks with complex structures; for neural networks with few layers (such as the network in this paper), the closer the network gets to the optimization goal, the more likely it will oscillate, resulting in performance that does not meet the requirements.

### 2.4. Depression Classification Performance Evaluation Experiment

Classifier performance must be evaluated through a plethora of iterative tests. A total of 10 complete iterative processes were used for each replication experiment; these comprised a training phase (with five rounds of cross-validation) and a testing phase. The feature matrix is first randomized and divided into five parts: four for training data and one for validation data. The classifier's average performance is provided in terms of sensitivity, specificity, and accuracy after the training model is applied to the test set. The proposed method in this article is dependent on a partly connected neural network and a subconvolutional neural network. Subconvolutional neural networks' temporal complexity is first considered. Its temporal complexity is proportional to the number of network layers (*L*) and hidden neurons linked with them (*N*). In conclusion, this research illustrates IoT technology's immense promise in the realm of brain health care.

Figure 5 depicts the classifier's learning curve on the major depression dataset. A steady level of accuracy and no discernible delay can be seen in both the training and validation sets throughout the training period. On the other hand, a high degree of generalization is demonstrated by the classifier's excellent classification performance on the test set—it is able to screen for depression in this data set without over or under fitting.

Different classifiers were used to the same dataset (MPHC EEG data) for depressed state classification, and their classification performance metrics are provided in Table 1. Along with MLRW [8] this article implemented numerous exemplary neural network models, including Resnet-16 [19], CapsuleNet [20], and LeNet [21]. All of these classifiers were updated somewhat. The model's input (203232) and output dimensions (1), as well as the neural architecture's other hyperparameters and each layer, remain unchanged. The table indicates as follows: (1) the classifier suggested in this work is the best in all classification indices, and its high sensitivity and specificity demonstrate that it can successfully screen out not just depression sufferers but also normal individuals; (2) the classifier's performance. The findings show that the classifier can successfully describe the fundamental characteristics of depression by calculating entropy's information method clustering based division of neighbor propagation and assessing the CNN network's complexity in the depression classification job.

It is unrelated to the number of layers in the model's architecture. For instance, Resnet and CapsuleNet with more layers do not reach the required performance metrics but take significantly longer to train. This scenario might be explained by the classifier being very sophisticated. When significant data is omitted, over fitting occurs, leading in a decline in classification performance. How to improve the classifier's fit to the nonlinearity of different data sets will have a substantial impact on its performance, and understanding this difference requires an understanding of the neural network. One of the important challenges raised by the black box will be a primary focus of future study. The accuracy, sensitivity, and specificity of the proposed model are shown in Figures 6–8, respectively.

This group of experiments is aimed at shedding information on the pathological relationship between CNN and depression classification tasks. Classifier 1 was shown to better grasp how EEG data is processed by CNN due to its input being channel-related. Increase the level of activity as much as possible. A single channel is defined for each of the twenty activation matrices of size (3232) that correspond to the input layer's dimensions (20 (3232)). AP clustering is used to estimate the entropy's information for every activation matrix, and related results are subsequently projected onto a scalp topographic map. In addition, the average features of brain states linked with certain brain regions were illustrated in ten to twenty worldwide systems.

In the classification field, classifiers have a natural inclination to categories based on increasingly distinct qualities, which are generally deterministic. Random variables are characterized by their entropy, which is a measure of their ambiguity. The higher the information entropy, the more information is stored in the variable, and the more likely the variable is to survive. It is therefore possible to think of the process of solving classification problems in terms of decreasing uncertainty (complexity) in order to enhance entropy. Entropy is utilized to decide which activation matrices are employed by CNNs for categorization.

Figure 9 depicts the 3D scalp topography of the CNN based on the MPHC EEG data, channel-level (a) and brain region-level (b). Figure 9(a) shows that the entropy values of Cz, T3, T4, T6, and other channels are lower as compared to other channels, indicating that the classifier establishes the fundamental differentiation between depression and health using voltage-amplitude channels. There are considerable disparities in depressed pathways between the left and right temporal lobes as depicted by the three-dimensional scalp topographic map in Figure 9(b), which supports the data provider's pathological diagnosis [8].

## 3. Conclusion

On the severe public depression dataset, the approach suggested in this article achieves great classification accuracy: depression is distinguished with 99.08 percent accuracy, 98.77 percent sensitivity, and 99.42 percent specificity, outperforming previous methods. Additionally, by calculating entropy's information method clustering-based division of neighbor propagation and evaluating the CNN network's complexity in the depression classification task, the results demonstrate that the classifier can effectively describe the intrinsic characteristics of depression. The scope of this research is that the proposed method is implemented directly to the EEG data and may identify sad states correctly and fast without the requirement for processing or feature extraction. In experiments using publicly available data, the accuracy, sensitivity, and specificity of the healthy control group and the depression control group is calculated. Determining and comprehending if a neural network is providing correct predictions is a major task. In general, this study demonstrates the enormous potential of IoT technology in the field of brain health care. The clustering algorithm is not known a priori in the traditional cluster analysis technique. Rather, it iterates across each sample point's contesting cluster centers to maintain the best clustering quality. Without preprocessing or feature extraction, the method is applied directly to raw EEG data and is capable of correctly and rapidly identifying depressive states.

## Figures and Tables

**Figure 1:** System architecture.

**Figure 2:** Network structure of CNN.

**Figure 3:** Entropy's information calculation based on neighbor propagation clustering (a) and traditional (b).

**Figure 4:** Comparison curves of different optimization methods.

**Figure 5:** Training and validation process learning curve.

**Figure 6:** Comparative accuracy of proposed model.

**Figure 7:** Comparative sensitivity of proposed model.

**Figure 8:** Comparative specificity of proposed model.

**Figure 9:** Visualization of 3D scalp topography of convolution neural network at the channel level (a) and brain region level (b).

**Table 1:** Classification performance comparison of related methods.

Method	Accuracy/%	Sensitivity/%	Specificity/%	Time/min
MLRW	87.50	95.00	80.00	—
LeNet	94.55	94.57	94.52	2.8
Resnet-16	90.06	93.09	86.70	80.0
CapsuleNet	94.42	89.01	99.23	36.0
The method of this paper	99.08	98.77	99.42	3.0

## Data Availability

The data shall be made available on request.
